# Improved voltage scanning algorithm based MPPT algorithm for PV systems under partial shading conduction

**DOI:** 10.1016/j.heliyon.2024.e39382

**Published:** 2024-10-15

**Authors:** Resat Celikel, Musa Yilmaz, Ahmet Gundogdu

**Affiliations:** a Firat University, Technology Faculty, Department of Mechatronics, Elazig, Turkey; b Department of Electrical and Electronics Engineering, Batman University, Batman, 72100, Turkey; c Bourns College of Engineering, Center for Environmental Research and Technology, University of California at Riverside, Riverside, CA, 92521, USA

**Keywords:** Maximum power point tracking (MPPT), Voltage scanning algorithm, Voltage skipping algorithm, Partial shading conditions, Simulation studies

## Abstract

Maximum Power Point Tracking (MPPT) algorithms are crucial for maximizing power extraction from photovoltaic (PV) systems. Traditional MPPT methods often exhibit suboptimal performance under partial shading conditions. Hence, advanced MPPT algorithms have been developed to enhance efficiency in such scenarios. The voltage scanning-based MPPT algorithm is notable for its superior performance under partial shading, characterized by high tracking speed and efficiency. This study introduces a novel enhancement to this method—namely, a voltage skipping algorithm designed to further improve tracking speed. Unlike conventional scanning techniques, this approach dynamically calculates skipping voltages during operation, eliminating the need for prior knowledge of PV panel characteristics. Performance evaluation was conducted using a MATLAB/Simulink model of a PV system comprising 4 series panels and a boost converter, subjected to simulations under 5 distinct partial shading scenarios. Comparative analyses with established optimization algorithms such as particle swarm optimization, cuckoo search algorithm, and grey wolf optimization highlight the proposed method's effectiveness in terms of tracking speed and maximum power output. The proposed algorithm has worked with high efficiency of 99.28 %, 99.61 %, 99.13 %, 99.16 % and 99.58 % in 5 different scenarios, respectively. By using the proposed method, a significant superiority has been achieved over other methods, with tracking speeds of 0.26s, 0.22s, 0.2s, 0.22s and 0.26s, respectively.

## 1 Introduction

With increasing concerns over global warming and pollution caused by fossil fuels, there has been a growing interest in renewable energy sources. Solar energy plays a pivotal role in this transition, where Photovoltaic (PV) Systems are utilized to convert solar energy into electrical power. However, the efficiency of these systems remains a challenge. To maximize energy extraction from PV systems, Maximum Power Point Tracking (MPPT) algorithms are crucial [1,2]. Among them, Perturb & Observe (P&O) and Incremental Conductance (InC) are widely adopted but struggle under partial shading conditions [3]. Recently, new MPPT algorithms leveraging fuzzy logic and artificial intelligence have emerged, demonstrating robust performance across various scenarios and actual radiation conditions [[4], [5], [6]].

Partial Shading Conditions (PSC) significantly affect the maximum power output of PV systems, posing a challenge that traditional methods often fail to address. Optimization algorithms, however, provide substantial advantages in identifying the Maximum Power Point (MPP). Among these optimization methods, the Particle Swarm Optimization (PSO) method has gained considerable attention in optimizing PV systems under PSC. Liu et al. implemented a PSO-based MPPT method to achieve peak power from PV panels under partial shading [7]. Renaudineau et al. utilized PSO to maximize power in a grid-connected PV system operating under varying environmental conditions [8]. Ishaque et al. improved steady-state performance by integrating PSO with the InC method [9]. Other studies have explored adaptations like dormant PSO, distribution-PSO, adaptive PSO, and modified PSO, each enhancing efficiency and tracking speed [[10], [11], [12], [13]]. Hybrid approaches combining PSO with P&O have also shown promise in optimizing PV systems for both uniform sunlight and PSC [14].

The Cuckoo Search Algorithm (CSA), initially introduced as a general optimization tool in 2009, has also found application in MPPT for PV systems [15]. Ahmed et al. compared CSA with traditional methods like P&O and PSO, highlighting its superior performance [16]. CSA variants, often integrating with the Levy flight algorithm, have been developed to increase computational efficiency [17,18]. Recent studies have simplified and enhanced CSA-based MPPT algorithms to achieve higher efficiency and improved duty cycle calculations [[19], [20], [21]].

Grey Wolf Optimization (GWO) and its variants have emerged as another effective approach for MPPT under PSC [22]. Mohanty et al. devised a hybrid GWO method combining P&O to enhance efficiency and tracking speed [23]. Comparative studies have shown GWO's superiority over traditional methods, emphasizing its robustness and efficiency gains [24,25]. Applications of GWO-based MPPT extend to grid-connected PV systems, focusing on maximizing system efficiency [26]. The salp swarm algorithm and the GWO method were used together in a high-efficiency hybrid MPPT algorithm, which was formed by combining two different optimization methods [27]. Diğer bir calısmada PV sistemin DC empedans karekteristiği cıkartılarak GWO yöntemi ile beraber kullanılarak MPPT algoritması geliştirlmiştir. In another study, the DC impedance characteristic of the PV system was extracted and the MPPT algorithm was developed using the GWO method [28]. By using a GWO algorithm modified in Ref. [29], power could be obtained from the PV system with both high speed and high efficiency.

In the control of PV systems, controller parameters are calculated using different optimization methods. These controllers are newer optimization algorithms such as emperor penguin optimizer (EPO) and the cuttlefish algorithm (CFA) that work with higher performance, as well as old optimization methods such as PSO [[30], [31], [32]].

Voltage scanning (VSC) and segmentation algorithms are pivotal for optimizing PV systems under varying shading conditions [33]. Recent advancements include duty cycle and voltage scanning algorithms by Başoğlu, innovative MPPT methods by Jately utilizing dynamic scanning techniques, and high-efficiency approaches by Kesilmiş detecting voltage breakpoints [[34], [35], [36], [37]]. VSC and spline-based methods have further improved MPPT performance under partial shading conditions [38,39]. Lyden et al. combined Simulated Annealing with voltage scanning to develop efficient MPPT solutions [40].

Zhang et al. formulated a hybrid MPPT algorithm integrating voltage scanning with artificial neural networks (ANN), demonstrating superior performance in simulations [41]. Another recent study introduced a voltage scanning algorithm that accelerates operation by selectively skipping voltage ranges, thus enhancing efficiency [40]. When analyzing voltage scanning or segmentation algorithms, it is apparent that the number of panels and voltage levels must be known. Different values are required for different PV systems. High efficiency can only be achieved using hybrid algorithms to adapt to changes in PV panel parameters over time. Source [38] shows the development of an adaptive voltage scanning-based MPPT algorithm to address these issues.

An adaptive skipping algorithm is given in Ref. [42]. This algorithm is used with the P&O method. In this algorithm, panel data is used for the screening process and for the detection of PSC status. However, in the proposed method, panel data is not required for the screening process. In the skipping algorithm given in Ref. [43], each voltage region is found under PSC conditions by using panel data. For this, the open circuit voltage of the system and the number of series connected panels are needed. However, the proposed algorithm does not use the data of the panels. The data of the panels may not be exactly the same during production or may differ over time according to the environmental conditions. The proposed algorithm eliminates this disadvantage. In addition, the proposed algorithm has a simpler structure. Because [42,43] also use the P&O algorithm. A similar method is used in Ref. [44], but this method also has an additional dependence on panel data. In Ref. [45], a skipping algorithm was developed to enhance the algorithm's speed, but the skipping voltage was approximated by inputting a specific value, which varies for each PV system. The most important disadvantage of this method is that it calls and runs different subalgorithms for three different situations while finding the GMPP point, which increases the processing intensity.

The proposed study developed a voltage scanning method and a skipping algorithm to increase speed without requiring information about panel voltage or skipping voltage, and the proposed algorithm has a simple structure. In this study, the simulation of optimization-based PSO, CSA, and GWO-based MPPT methods, as well as voltage scanning (VSC) and proposed methods (VSC-Skipping), was performed in the MATLAB/Simulink environment for a PV system operating under PSC, consisting of 4 series panels and a DC-DC boost converter. These algorithms were tested under five different PSCs in the MATLAB/Simulink environment. The simulation results were thoroughly examined, comparing the efficiencies and tracking speeds of the algorithms, and the findings were interpreted.

## 2 PV system modeling

PV system modeling involves constructing electrical equivalent circuit models of photovoltaic (PV) cells and expressing these models mathematically. Fig. 1 depicts the electrical equivalent circuit model of a PV cell, including resistors, a diode, and a current source. The expression of the current to be obtained from a PV cell is given in detail in Ref. [3].

**Fig. 1:** Equivalent circuit model of the PV cell.

In this context, parameters describing the PV cell, where Equation (4) specifies the current generated under standard conditions of 25 °C and 1000 W/m^2^.

Fig. 2 illustrates a PV string under uniform sunlight (Fig. 2a) and partial shading conditions (Fig. 2b). The impact of partial shading conditions on the PV system's power output and maximum power point voltage is evident, highlighting the limitations of traditional MPPT methods for such conditions. PV system modeling is crucial for understanding PV system behavior under varying solar radiation and environmental conditions, aiding in system design, optimization, and performance prediction.

**Fig. 2:** PV string a) Uniform sunlight b) Partial shading.

## 3 Optimization and voltage scanning based MPPT methods

Among the methods used to extract maximum power from PV power systems operating under PSC, optimization methods are increasingly maintaining their relevance. The primary goal in developing optimization methods is to ensure the extraction of maximum power and to achieve this extraction in the shortest possible time. This study examines some of the most widely used methods, including PSO, CSA, and GWO. Additionally, the results obtained using VSC and VSC-Skipping algorithms are compared with these methods.

### 3.1 PSO-based MPPT method

The PSO method is an optimization algorithm inspired by the collective behavior of flocks of birds and schools of fish. In this algorithm, particles, representing agents, exchange information during their search for optimal solutions. Each particle follows two rules: it adjusts its position towards its personal best (p_best,i) and the global best position (g_best), found by any particle in the swarm.

This iterative process enables particles to converge towards an optimal or near-optimal solution. The standard PSO equations are defined as follows [7]:

(1) $$v_{i}\left(k+1\right)=wv_{i}\left(k\right)+c_{1}r_{1}.\left(p_{best,i}-x_{i}\left(k\right)\right)+c_{2}r_{2}.\left(g_{best}-x_{i}\left(k\right)\right)$$

(2) $$x_{i}\left(k+1\right)=x_{i}\left(k\right)+v_{i}\left(k+1\right),i=1,2,\ldots \ldots \ldots N$$

The flowchart illustrating the PSO-based MPPT method is presented in Fig. 3.

**Fig. 3:** Flowchart of the PSO-based MPPT method.

### 3.2 CSA-based MPPT method

The Cuckoo Search Algorithm (CSA) operates based on three core principles. Firstly, in each iteration, every cuckoo lays one egg and then selects a random nest to deposit this egg. This process generates a duty cycle D at each iteration. Secondly, the nest with the best egg is retained and carried over to the next generation, representing the optimal duty cycle for subsequent iterations. Thirdly, with a probability pa ∈ [0, 1], a host bird may discover a foreign egg. In response, the MPPT algorithm discards the duty cycle associated with the lowest power value and replaces it with a new duty cycle. The new duty cycle is generated using the Levy flight equation, shown in Equation (3).

(3) $$D_{i}^{t+1}=D_{i}^{t}+\alpha ⊕le^{\prime }vy\left(\lambda \right),i=1,2,\ldots ..n$$

Here, n represents the problem size, and α is defined as in Equation (4). The symbol ⊕ denotes multiplication from an input perspective, and Levy(.) denotes a random walk drawn from a Levy distribution for step length, simplified in Equation (5).

(4) $$\alpha =\alpha_{0}\left(D_{best}-D_{i}\right)$$

(5) $$\alpha =\alpha_{0}\left(D_{best}-D_{i}\right)⊕le^{\prime }vy\left(\lambda \right)\approx k\times \left(\frac{u}{{\left|v\right|}^{\frac{1}{\beta }}}\right)\left(D_{best}-D_{i}\right)$$

Here, *β* = *1.5, k* is a coefficient chosen by the designer, *u* and *v* are normal distribution curves, and $\sigma_{u}$ and $\sigma_{u}$ are calculated as in equations (6), (7)).

(6) $$u\approx N\left(0,\sigma_{u}^{2}\right),v\approx N\left(0,\sigma_{v}^{2}\right)$$

(7) $$\sigma_{v}=1,\sigma_{v}=\left(\frac{\Gamma \left(1+\beta \right)\times \sin\;\left(\pi +\beta \backslash /2\right)}{\Gamma \left(1+\beta /2\right)\times \beta \times 2^{\left(\left(\beta -1\right)/2\right)}}\right)$$

The flowchart illustrating the operation of the CSA algorithm can be observed in Fig. 4.

**Fig. 4:** Flowchart of the CSA-Based MPPT method.

### 3.3 GWO-based MPPT method

Grey wolves, residing atop the food chain, thrive in packs. To mimic their leadership structure, the Grey Wolf Optimizer (GWO) employs four types: alpha (α), beta (β), delta (δ), and omega (ω). Alpha (α) symbolizes the optimal solution, reflecting the wolves' hierarchical organization. Beta (β) and delta (δ) denote the second and third best solutions, respectively, while omega (ω) represents all other candidate solutions. During hunting, grey wolves exhibit encircling behavior around their prey, which is mathematically modeled through the following equations:

(8) $$\vec{D}=\left|\vec{C}.{\vec{X}}_{p}\left(t\right)-{\vec{X}}_{p}\left(t\right)\right|$$

(9) $$\vec{X}\left(t+1\right)=\left|{\vec{X}}_{p}\left(t\right)-\vec{A.}\vec{D}\right|$$

(10) $$\vec{A}=2\vec{a}.{\vec{r}}_{1}-\vec{a}$$

(11) $$\vec{C}=2{\vec{.r}}_{2}$$

(12) $$D\left(k+1\right)=D_{i}\left(k\right)-A.D$$

(13) $$P\left(d_{i}^{k}\right)>\;P\left(d_{i}^{k-1}\right)$$

The flowchart of the GWO algorithm's operation can be seen in Fig. 5.

**Fig. 5:** Flowchart of the GWO-Based MPPT method.

### 3.4 VSC-skipping MPPT algorithm

The VSC-Skipping MPPT Algorithm, represents a significant advancement in scanning-based MPPT methodologies. These algorithms are extensively documented in the literature for their efficacy in optimizing PV system performance under varying conditions. Specifically, the Voltage Scanning (VSC) algorithm incrementally adjusts the voltage and identifies the corresponding maximum power points. Fig. 6 illustrates the procedural flow of the proposed algorithm, highlighting its sequential steps and decision points. Equation (14) defines the formulation for the linear increase in reference voltage, a critical component in the algorithm's execution and optimization process.

(14) $$V_{\ln\;\_r}=V_{i}+\Delta V_{i}$$

Here, $V_{\ln\;\_r}$ represents the linearly increasing reference voltage, $V_{i}$ represents the initial voltage, and $\Delta V_{i}$ represents the voltage increment. It is important that the value of $\Delta V_{i}$ is not chosen too high to prevent the voltage reference from increasing uncontrollably. As the voltage reference increases, changes in power and voltage on the panel are also detected, as seen in Equation 15.

(15) $$\Delta V=V_{n}-V_{\left(n+1\right)}\;and\Delta P=P_{n}-P_{\left(n+1\right)}$$

When the power difference ΔP is less than 0.001, power and voltage samples are taken. The higher power sample is identified as the Greater Maximum Power Point (GMPP) compared to the previous maximum. If the system voltage approaches the last possible value, V_oc_, this indicates that the scanning process must be terminated. Here, 0.9∗V_oc_ data is used to complete the scanning process. This value is not a definite and necessarily correct value. An approximate value will be sufficient to complete the scanning. In fact, the output voltage value of the known PV system will again be approximately sufficient. Subsequently, when both |ΔP| and and |ΔV| are less than 0.001, the voltage at the GMPP becomes the reference voltage, ending the scanning process. The PV system's voltage is adjusted to match this reference, while skipping voltages, calculated using Equation (16), are gradually added to the increasing reference voltage to ensure smooth adjustments. Fig. 7 illustrates these voltage regions and skipping voltage calculations for a PV system under PSC5.

(16) $$\left\{\begin{array}{c} V_{\ln\;\_r}=V_{ref}+V_{ref1}+V_{ref2}+V_{ref3}+\ldots \ldots \ldots +V_{refn}\\ V_{ref1}=V_{ref}+V_{s}\\ V_{ref2}=V_{ref1}+V_{s1}\\ V_{ref3}=V_{ref2}+V_{s2}\\ V_{ref\left(n\right)}=V_{ref\left(n-1\right)}+V_{s\left(n-1\right)} \end{array}\right\}$$

Here, $V_{s}$ is calculated separately for each region and added to the previous reference voltage. In traditional skipping algorithms, this voltage is obtained from the data of the panels in the system or estimated approximately. In the MPPT algorithm implemented in this study, $V_{s}$ is calculated separately at each maximum power region without the need for panel information. This allows the algorithm to work without panel information in different systems. Additionally, by calculating the skipping voltage and adding it to the scanning voltage, the operation speed of MPPT can be increased without being affected by changing parameters over long periods of use.

**Fig. 6:** Flowchart of the VSC-skipping MPPT algorithm.

**Fig. 7:** Skipping voltage and maximum power regions in a PV system operating under PSC5.

## 4 Simulation and results

To test the proposed algorithm, a PV system has been created in the MATLAB/Simulink environment. In this simulation, there are four series-connected panels and a DC-DC boost converter connected to these panels. The input side capacitance of the boost converter is C_1_ = 10 μF, the output side capacitance is C = 467 μF and the inductance is L = 1.15 mH. The model of the panels used is Tata Power, with the code TP250MBZ. The parameters of the panel are given in Table 1.

**Table 1:** Parameters of Tata power TP250MBZ.

**PV MODULE (SPR-415E-WHT-D)**	Symbol	Quantity	Values	
	*P*_*MPP*_	Maximum power at MPP	249	W
	*V*_*MPP*_	Voltage at MPP	30	V
	*I*_*MPP*_	Current at MPP	8.3	A
	*V*_*OC*_	Open-circuit voltage	36.8	V
	*I*_*SC*_	Short-circuit current	8.83	A
	*T*_*C*_	Temp. Coefficient of Voc	−0.33	%/^ο^C
	*T*_*C*_	Temp. Coefficient of Isc	0.063805	%/^ο^C
	*R*_*S*_	Series res. of PV cell	0.2914	Ω
	*R*_*P*_	Shunt res. of PV cell	314.7646	Ω
	*N*_*cell*_	Cells per module	60	

Under nominal test conditions, the maximum power that each panel can generate is 249W, and the voltage value at maximum power is given as 30V. Five different scenarios have been created to measure the performance of PSO, CSA, GWO, VSC, and VSC-Skipping algorithms. These scenarios are shown in Fig. 8. Accordingly, in the created PSC scenarios, different power values are present at different voltage values.

**Fig. 8:** Partially different PSCs and GMPPs created in the PV system.

In MATLAB simulation, a 50 kHz switching frequency is chosen for the DC-DC converter. Current and voltage readings from the PV panel are used to compute power values in the MPPT algorithm, which determines the switching intervals for the boost converter. Fig. 9 depicts the schematic diagram of the PV power system developed in the MATLAB/Simulink environment.

**Fig. 9:** PV power system created in MATLAB/Simulink Workspace.

The power values and duty cycles obtained from the simulation results were analyzed in detail. Accordingly, Fig. 10 shows the maximum power obtained from the PV system operating under PSC1 for 5 different MPPT algorithms.

**Fig. 10:** Powers obtained from the PV system operating under PSC1 using PSO, CSA, GWO, VSC, and VSC-skipping algorithms.

As seen in Fig. 10, the VSC-Skipping method achieves the maximum power point in a very short time, such as 0.26s, with very high performance. The highest power value produced is obtained by the CSA method, at 637.8 W. In addition, the VSC and VSC-Skipping methods produce 634.8W of power, approaching this power value closely.

Fig. 11 shows the maximum powers obtained from the PV system operating under PSC2 for five different MPPT algorithms. Under these conditions, it can be seen that the VSC-Skipping algorithm produces the maximum power in the shortest time. The maximum power produced is 409.6W. The tracking speed of the algorithm is 0.22s.

**Fig. 11:** Powers obtained from the PV system operating under PSC2 using PSO, CSA, GWO, VSC, and VSC-skipping algorithms.

Fig. 12 shows the maximum powers obtained from the PV system operating under PSC3 for five different MPPT algorithms. Under these conditions, it can be seen that the VSC and VSC-Skipping algorithms produce the highest power (228.8W) in the shortest time (0.2s). The superiority of the VSC and VSC-Skipping algorithms over the other algorithms is clearly evident under these conditions.

**Fig. 12:** Powers obtained from the PV system operating under PSC3 using PSO, CSA, GWO, VSC, and VSC-skipping algorithms.

In Fig. 13, the maximum powers obtained from the PV system operating under PSC4 for five different MPPT algorithms are shown. Under these conditions, it can be seen that the VSC and VSC-Skipping algorithms produce the highest power (206.65W) in the shortest time (0.22s).

**Fig. 13:** Powers obtained from the PV system operating under PSC4 using PSO, CSA, GWO, VSC, and VSC-skipping algorithms.

In Fig. 14, it is observed that the largest power obtained from the PV system operating under PSC5 is 760.7W with the VSC algorithm. The power generated by the VSC-Skipping algorithm is very close to this value at 759.5W. On the other hand, the VSC-Skipping algorithm has the highest tracking speed at 0.26s.

**Fig. 14:** Powers obtained from the PV system operating under PSC5 using PSO, CSA, GWO, VSC, and VSC-skipping algorithms.

Table 2 shows detailed data on the results obtained with all scenarios and MPPT methods. According to this table, at the lowest voltage levels where maximum power values occur (PSC3-PSC4), both VSC and VSC-Skipping algorithms have shown the same performance and have provided a significant advantage over other MPPT algorithms in terms of both power values and tracking speeds. Additionally, under PSC4, optimization algorithms have deviated significantly from the maximum power value. In all scenarios, the highest tracking speed has been achieved using the VSC-Skipping algorithm. It is observed that optimization algorithms have very low tracking speeds. While VSC-Skipping and VSC algorithms produce approximately the same power in the average of the five scenarios, optimization algorithms have reached lower power averages. Consequently, when the table values are examined in detail, it is clearly seen that the VSC-Skipping algorithm has the highest tracking speed and has a clear advantage over the VSC algorithm in this respect.

**Table 2:** Performance of five different MPPT methods in a PV system operating under five different scenarios.

GMPP (W)		Max. Power (W)	MPP Voltage (V)	Track. Eff. (%)	Track. Speed(s)	Cov. Time (s)
PSC1 639.4W 93.1V	**PSO**	636	94	99.46	>3	1.5
	**CSA**	**637.8**	93.05	99.74	0.9	0.5
	**GWO**	634	94.4	99.21	0.7	0.6
	**VSC**	634.8	93.2	99.28	0.33	0.3
	**VSC-Skipping**	634.8	93.4	99.28	**0.26**	**0.25**
PSC2 411.2W 60.4V	**PSO**	406	61.7	98.73	>3	>3
	**CSA**	408.35	61	99.3	2.8	1
	**GWO**	409.5	60.45	99.58	0.8	0.7
	**VSC**	409.3	60.6	99.53	0.26	0.23
	**VSC-Skipping**	**409.6**	60.12	99.61	**0.22**	**0.2**
PSC3 230.8W 27.8V	**PSO**	224	28.7	97.05	>3	>3
	**CSA**	215.2	29.7	93.24	2.5	1.6
	**GWO**	209.6	30	90.81	0.8	0.7
	**VSC**	**228.8**	27.9	99.13	0.2	0.17
	**VSC-Skipping**	**228.8**	27.9	99.13	**0.2**	**0.17**
PSC4 208.4W 28V	**PSO**	160.2	62.5	76.87	>3	1.5
	**CSA**	160.2	62.5	76.87	1.5	0.95
	**GWO**	159.4	61.5	76.48	0.8	0.6
	**VSC**	**206.65**	27.95	99.16	0.22	0.165
	**VSC-Skipping**	**206.65**	27.95	99.16	**0.22**	**0.155**
PSC5 762.7W 126.3V	**PSO**	760.5	126.8	99.71	>3	1.8
	**CSA**	760.2	125.2	99.67	1	1.5
	**GWO**	733	130.2	96.1	0.65	0.54
	**VSC**	**760.7**	126.4	99.73	0.28	0.27
	**VSC-Skipping**	759.5	127.5	99.58	**0.26**	**0.25**

In Fig. 15, the duty cycles generated by five different MPPT methods for each scenario are shown. It is evident that optimization algorithms lag significantly in capturing the maximum power point. On the other hand, it can be seen that the speed of the VSC-Skipping algorithm is higher than the VSC algorithm, except for PSC3-PSC4, where it is approximately the same.

**Fig. 15:** Duty cycles for PSO, CSA, GWO, VSC, and VSC-skipping algorithms for 5 different scenarios.

In Fig. 16, Figure 17, the PV system voltages and currents generated by each MPPT algorithm under each shading condition are shown, respectively.

**Fig. 16:** Voltages for PSO, CSA, GWO, VSC, and VSC-skipping algorithms for 5 different scenarios.

**Figure 17:** Currents for PSO, CSA, GWO, VSC, and VSC-skipping algorithms for 5 different scenarios.

In Fig. 18, a comparison of the speeds of the VSC and VSC-Skipping algorithms can be made. It is clearly seen that the speed of the proposed algorithm is high in all scenarios except PSC3. In the PSC3 scenario, the operating speeds of both algorithms are the same. The tracking speeds and efficiencies of the algorithms are detailed in Table 1.

**Fig. 18:** MPPT speeds of VSC and VSC-skipping algorithms for 5 different scenarios.

The proposed algorithm stands out with its high speed when compared to optimization algorithms. It is also seen that it works faster than the VSC method in almost all scenarios. On the other hand, except for scenario 1, it has managed to obtain more power in optimization methods in all other scenarios. In the study under PSC1, it has managed to obtain a value very close to the CSA algorithm. When the average of the efficiencies obtained in all PSC cases is taken, the average efficiency of the proposed method is 99.352 %, while the average speed is obtained as 0.232s. The average speed is obtained as 0.258s in the VSC algorithm, which works at the speed closest to the proposed algorithm.

## 5 Conclusion

In photovoltaic (PV) systems, various maximum power point tracking (MPPT) methods are used to achieve maximum power under partial shading conditions. These methods are expected to attain the highest power in the shortest time possible. In this study, a voltage scanning-based MPPT algorithm incorporating a highly efficient and fast skipping algorithm was developed. The algorithms were tested using a PV system created in MATLAB/Simulink under five different partial shading scenarios. The proposed algorithm was compared with the traditional voltage scanning control (VSC) algorithm along with particle swarm optimization (PSO), cuckoo search algorithm (CSA), and grey wolf optimization (GWO) algorithms. The VSC-Skipping algorithm, when averaged across the five scenarios, produced approximately the same power as the VSC method, with 448.05W and 447.81W, respectively. These power values demonstrate significant superiority of scanning methods over other methods. Considering the tracking speed, the VSC-Skipping algorithm is the fastest, achieving a tracking speed of 0.232s on average across the five scenarios. The closest tracking speed value is obtained with the VSC algorithm, at 0.258s. The VSC and VSC-Skipping algorithms, particularly in capturing maximum power values at low voltage levels, have shown significant advantages over other methods.

On the other hand, traditional scanning algorithms and voltage division algorithms, such as those based on 0.8Voc, require PV panel data. The proposed algorithm can operate without the need for panel data and is not affected by changing panel parameters during operation. This is because it independently scans the panel data and calculates the skipping voltage during scanning.

In future studies, the voltage increment value will be implemented adaptively rather than linearly, aiming to further enhance MPPT efficiency. The adaptive voltage increment will be such that the initial increment will decrease as the high LMPP point is approached. This will be repeated in each region. This increment will be done using smart methods. Thus, reaching the GMPP point will be much faster. Additionally, advanced controller structures will be used to improve control performance, thereby minimizing access time to steady state and steady-state errors. The most important disadvantage of this method is that the voltage controller performance greatly affects the system performance and the noise that will occur in a real system will have an effect on the measurement. For this reason, a very good filtering is necessary in the measurement.

## CRediT authorship contribution statement

**Resat Celikel:** Writing – original draft, Investigation, Formal analysis, Conceptualization. **Musa Yilmaz:** Writing – review & editing, Validation, Supervision, Methodology. **Ahmet Gundogdu:** Writing – original draft, Validation, Software, Methodology.

## Declaration of competing interest

The authors declare that they have no known competing financial interests or personal relationships that could have appeared to influence the work reported in this paper.
